The article "To Analyze the Influencing Factors of Senile Coronary Heart Disease Patients Complicated with Frailty Syndrome" was retracted in 2023. Reasons: signs of a paper mill; suspected computer-generated content; unreliable results or conclusions; concerns about the data.

# To Analyze the Influencing Factors of Senile Coronary Heart Disease Patients Complicated with Frailty Syndrome

**DOI:** 10.1155/2022/7619438

**Published:** 2022-01-07

**Authors:** Tian Qin, Wang Sheng, Guoheng Hu

**Affiliations:** ^1^Hunan University of Chinese Medicine, Changsha 410000, China; ^2^The Second Hospital of Hunan University of Chinese Medicine, Changsha 410000, China; ^3^The First Hospital of Hunan University of Chinese Medicine, Changsha 410000, China

## Abstract

To analyze the influencing factors of senile coronary heart disease patients complicated with frailty syndrome. A total of 80 elderly patients with coronary heart disease admitted to our hospital from March 2020 to March 2021 were selected as the research subjects. The Fried Frailty Symptom Scale was used to evaluate whether the 80 patients were complicated with frailty syndrome. According to the evaluation results, the patients were divided into a nonfrailty syndrome group (52 cases in total) and frailty syndrome group (28 cases in total). Clinical data of two groups of patients were collected, and multivariate logistic regression was used to analyze the influencing factors of senile coronary heart disease patients complicated with frailty syndrome. Among 80 patients, the incidence of frailty syndrome was 35.00% (28/80), including 18 cases in early frailty and 10 cases in frailty stage. Univariate analysis showed that age, body mass (BMI), diabetes mellitus, congestive heart failure, chronic renal insufficiency, chronic obstructive pulmonary disease (COPD), tumor, high uric acid hematic disease, arrhythmia, interleukin-6 (IL-6), c-reactive protein (CRP), fibrinogen (FIB), brain natriuretic peptide (BNP), uric acid (UA), serum creatinine (Scr), serum protein (ALB), white blood cell count (WBC), and neutrophil count were the possible risk factors for senile coronary heart disease complicated with frailty syndrome (*P* < 0.05). Multivariate logistic regression analysis showed that combined COPD, combined tumor, IL-6, BNP, UA, SCR, ALB, and neutrophil count were independent risk factors for senile CHD complicated with frailty syndrome (*P* < 0.05). Combined with COPD, combined with tumor, IL-6, BNP, UA, SCR, ALB, and neutron cell count are the influencing factors for senile coronary heart disease patients complicated with frailty syndrome. These factors can be used as the basis for the diagnosis of frailty syndrome and guide the clinical development of targeted diagnosis and treatment plan.

## 1. Introduction

Coronary heart disease mainly refers to the abnormal lipid metabolism. The lipids in the blood deposit on the smooth arterial intima. The accumulation of atheroma-like lipids in the arterial intima leads to the formation of white plaques. As the plaques gradually increase, it can cause arterial stenosis, block blood flow, and heart ischemia and induce angina pectoris [1–3]. In recent years, with the increasing aging of our society, the clinical incidence of coronary heart disease is getting higher and higher, and it has become a major disease threatening the health of the elderly [4]. For patients with coronary heart disease, their functional status will have a great impact on treatment and prognosis, and frailty syndrome is the main manifestation of reduced functional status. Frailty syndrome is a nonspecific state in which the physiological reserve of the elderly decreases, increases the vulnerability of the body, and weakens the body's ability to resist stress [5, 6]. In recent years, studies have gradually begun to explore the relevant influencing factors of elderly coronary heart disease complicated by frailty syndrome and to predict the patient's condition in a timely manner. In view of this, this study selected 80 elderly patients with coronary heart disease admitted in our hospital from March 2020 to March 2021 as the research objects, aiming to analyze the influencing factors of elderly coronary heart disease patients with debilitating syndrome.

The article "To Analyze the Influencing Factors of Senile Coronary Heart Disease Patients Complicated with Frailty Syndrome" was retracted in 2023. Reasons: signs of a paper mill; suspected computer-generated content; unreliable results or conclusions; concerns about the data.

## 2. Materials and Methods

### 2.1. General Information

We selected 80 elderly patients with coronary heart disease accepted by our hospital from March 2020 to March 2021 as the subjects of this study. The Fried Debilitating Symptom Scale was used to assess whether the 80 patients were associated with debilitating syndromes, and the patients were classified as noncombined patients based on the evaluation results.

#### 2.1.1. Inclusion Criteria

- Coronary angiography showed that one or more coronary arteries had stenosis ≥50%
- Age ≥60 years
- Complete clinical data
- Patients and their family members were aware of the study and had already signed the informed consent form

#### 2.1.2. Exclusion Criteria

- Patients with malignant tumors.
- Patients with hematological diseases or systemic infectious diseases.
- Patients who refuse to cooperate with debilitating examinations.
- Patients with history of mental illness or cognitive dysfunction. The study has been approved by the ethics committee of the hospital.

### 2.2. Methods

The “Fried Debilitating Symptom Scale” was used to evaluate the debilitating condition of 80 patients. The evaluation content included fatigue, decreased BMI, weakness, decreased walking speed, and decreased physical activity. If none of the above exists, it is a nondebilitating period, with 1-2 items in the predebility period and 3 items and above in the debility period. According to the evaluation results, 80 patients were divided into a nondebilitating syndrome group and debilitating syndrome group (including predebility and debilitating period).

The article "To Analyze the Influencing Factors of Senile Coronary Heart Disease Patients Complicated with Frailty Syndrome" was retracted in 2023. Reasons: signs of a paper mill; suspected computer-generated content; unreliable results or conclusions; concerns about the data.

The clinical data of 80 patients were collected, and the “general information questionnaire” designed by our hospital was used for investigation, which included the patient's name, gender, age, body mass (BMI), smoking history (previous smoking for six months or more) and drinking history (previous drinking for half a year or more), and combined diseases (hypertension, diabetes, congestive heart failure, chronic renal insufficiency, chronic obstructive pulmonary disease (COPD), tumor, hyperuricemia, arrhythmia, and cerebrovascular disease).

80 patients were tested for laboratory indicators: 5 mL of fasting venous blood was collected from the patients in the morning, and the blood samples were tested by the inspectors of the laboratory of our hospital. The measurement indicators mainly include interleukin-6 (IL-6), procalcitonin (PCT), C-reactive protein (CRP), D-dimer (DD), fibrinogen (FIB), brain natriuretic peptide (BNP), uric acid (UA), serum creatinine (Scr), serum albumin (ALB), total cholesterol (TC), triacylglycerol (TG), low-density lipoprotein cholesterol (LDL-C), high-density lipoprotein cholesterol (HDL-C), hemoglobin (Hb), white blood cell count (WBC), and neutrophil count.

### 2.3. Statistical Methods

SPSS 22.0 statistical software was used for data analysis. Measurement data conforming to the normal distribution were expressed as mean ± standard deviation ($\bar{x}\pm s$). The comparison between the two groups was performed by the *t*-test. Those who did not conform to the normal distribution were converted to normal distribution and then counted. Scientific analysis: counting data were expressed by rate, and comparison between groups was performed by the *χ*2 test; multivariate analysis was conducted by logistic regression analysis; *P* < 0.05 was considered as the statistically significant difference.

## 3. Results

After evaluation, it was found that 80 patients had 28 cases of debilitating syndrome, with an incidence rate of 35.00%, of which 18 were in the predebilitating stage and 10 were in the debilitating stage. As shown in Table 1, there was no significant difference between the two groups in terms of gender, smoking history, drinking history, hypertension, and cerebrovascular disease (*P* > 0.05); in terms of age, BMI, diabetes, congestive heart failure, chronic renal insufficiency, COPD, tumor, hyperuricemia, and arrhythmia, the difference between the two groups was statistically significant (*P* < 0.05). Table 1 shows the comparison of general information between the nondebilitating syndrome group and the debilitating syndrome group.

The article "To Analyze the Influencing Factors of Senile Coronary Heart Disease Patients Complicated with Frailty Syndrome" was retracted in 2023. Reasons: signs of a paper mill; suspected computer-generated content; unreliable results or conclusions; concerns about the data.

The levels of PCT, DD, TC, TG, LDL-C, HDL-C, and Hb in the two groups were similar, and the difference was not statistically significant (*P* > 0.05); IL-6, CRP, FIB, BNP, UA, Scr, WBC, and neutrophil count levels in the frailty syndrome group were higher than those in the nondebilitating syndrome group, and their ALB levels were lower than those in the nondebilitating syndrome group (*P* < 0.05).  Table 2 is the comparison of laboratory indicators between the two groups.  Figure 1 is the comparison of IL-6, Scr, and ALB levels between the two groups.  Figure 2 illustrates the comparison of CPR, FIB, WBC, and NC levels between the two groups.  Figure 3 shows the comparison of BNP and UA levels between the two groups.

Multivariate logistic regression analysis was carried out according to single-factor analysis in Tables 2 and 3. The results showed that the combined COPD, combined tumor, IL-6, BNP, UA, Scr, ALB, and neutrophil count are the combination of elderly patients with coronary heart disease combined with frailty independent risk factors for symptoms (*P* < 0.05).  Table 3 is the multivariate logistic regression analysis.

## 4. Discussion

Coronary heart disease is a common disease in the elderly. According to relevant statistics, the number of patients suffering from cardiovascular disease in our country is 290 million, of which 11 million are coronary heart disease, and the incidence of this disease is still on the rise in recent years [7]. In the elderly population, weakening of physical function is very common, and the decline of physical function is the main factor that causes weakness, and the occurrence of weakness is an important factor in predicting the poor prognosis of cardiovascular disease. According to relevant statistics, the incidence of frailty syndrome in elderly patients with coronary heart disease is as high as 48.5%–79.0% [8]. Therefore, the influencing factors of elderly coronary heart disease with frailty syndrome have become a hot spot in clinical research at this stage.

In this study, it was found that a total of 28 cases of frailty syndrome occurred in 80 patients, with an incidence rate of 35.00%. Frailty syndrome is more common in elderly patients with coronary heart disease. In terms of influencing factors, multivariate logistic regression analysis showed that combined COPD, combined tumor, IL-6, BNP, UA, Scr, ALB, and neutrophil count are independent risk factors for elderly coronary heart disease patients with frailty syndrome (*P* < 0.05). The specific analysis is as follows: The first is the combination of COPD and tumor: COPD is a lung disease characterized by airflow limitation. This disease will severely reduce the patient's lung function and weaken the physical function [9, 10]. The presence of tumors will seriously affect the various body functions of the patient, and it is also a major factor leading to the decline of body functions. In clinical practice, the combination of one of the abovementioned diseases will increase the risk of debilitating elderly patients with coronary heart disease [11]. Chatterjee et al. [12] believe that, for elderly patients with coronary heart disease, clinicians need to understand the status of their combined diseases in order to do a good job in the early screening of elderly patients with coronary heart disease and improve the prognosis of patients as much as possible. The second is laboratory indicators: this study found that IL-6, BNP, UA, Scr, ALB, and neutrophil count are one of the influencing factors of elderly coronary heart disease with frailty syndrome, so these indicators can be used as a clinical assessment of patient frailty-related laboratory indicators. The reason is that the subclinical and comorbidities of elderly patients with coronary heart disease will reduce their systemic physiological reserves, reduce body balance, and cause significant changes in the abovementioned laboratory indicators [13–15]. However, in the study of Stewart et al. [16], the univariate analysis believed that BNP and Scr were possible influencing factors in elderly patients with coronary heart disease, but multivariate logistic regression analysis showed that BNP and Scr could not be influencing factors. There is a certain difference between this result and the results of this study, which may be related to factors such as individual differences in patients and differences in the sample size of the study. In short, for elderly patients with coronary heart disease, the overall reserve function status of the patient can be assessed based on the abovementioned related influencing factors, so as to accurately screen the occurrence of debilitating syndrome early and improve the patient's prognosis [17]. The related research on elderly patients with coronary heart disease complicated by frailty syndrome is still in the preliminary stage, and the lack of large-scale epidemiological investigations has led to the lack of frailty scores or diagnostic models. After this study, the related factors of frailty can be further clarified, which is of great significance for constructing frailty scores or diagnostic models [18, 19].

The article "To Analyze the Influencing Factors of Senile Coronary Heart Disease Patients Complicated with Frailty Syndrome" was retracted in 2023. Reasons: signs of a paper mill; suspected computer-generated content; unreliable results or conclusions; concerns about the data.

## 5. Conclusions

In conclusion, combined COPD, combined tumor, IL-6, BNP, UA, Scr, ALB, and neutrophil count are the influencing factors of elderly patients with coronary heart disease combined with frailty syndrome, and these factors can be used as the basis for the diagnosis of frailty syndrome and to guide the clinical development of targeted diagnosis and treatment plans.

## Figures and Tables

**Figure 1:** Comparison of IL-6, Scr, and ALB levels between the two groups. *Note*. Compared with the nondebilitating syndrome group, ^*∗*^*P* < 0.05.

**Figure 2:** Comparison of CPR, FIB, WBC, and NC levels between the two groups. *Note*. Compared with the nondebilitating syndrome group, ^*∗*^*P* < 0.05.

**Figure 3:** Comparison of BNP and UA levels between the two groups. *Note*. Compared with the nondebilitating syndrome group, ^*∗*^*P* < 0.05.

**Table 1:** Comparison of general information between the nondebilitating syndrome group and the debilitating syndrome group (*n*, %).

Project		Nondebilitating syndrome group (*n* = 52)	Frailty syndrome group (*n* = 28)	*χ* ^2^	*P*
Gender	Male	27 (51.92)	17 (60.71)	0.568	0.451
	Female	25 (48.08)	11 (39.29)		

Age (years)	60–70	40 (76.92)	10 (35.71)	13.187	0.000
	＞70	12 (23.08)	18 (64.29)		

BMI (kg/m^2^)	≤24.5	37 (71.15)	8 (28.57)	13.410	0.000
	＞24.5	15 (28.85)	20 (71.43)		

History of smoking	Yes	30 (57.69)	17 (60.71)	0.069	0.793
	No	22 (42.31)	11 (39.29)		

History of drinking	Yes	31 (59.62)	18 (64.29)	0.167	0.683
	No	21 (40.38)	10 (35.71)		

Comorbidity	Hypertension	26 (50.00)	15 (53.57)	0.093	0.761
	Diabetes	18 (34.62)	17 (60.71)	5.038	0.025
	Congestive heart failure	18 (34.62)	18 (64.29)	6.474	0.011
	Chronic renal insufficiency	15 (28.85)	16 (57.14)	6.140	0.013
	COPD	13 (25.00)	20 (71.43)	16.189	0.000
	Tumor	5 (9.62)	15 (53.57)	18.755	0.000
	Hyperuricemia	3 (5.77)	14 (50.00)	21.277	0.000
	Arrhythmia	5 (9.62)	17 (60.71)	23.835	0.000
	Cerebrovascular disease	10 (19.23)	6 (21.43)	0.055	0.815

**Table 2:** Comparison of laboratory indicators between the two groups ($\bar{x}\pm s$).

Index	Nondebilitating syndrome group (*n* = 52)	Frailty syndrome group (*n* = 28)	*t* value	*P* value
IL-6 (ng/L)	10.28 ± 2.54	24.35 ± 3.19	17.252	0.000
PCT (*μ*g/L)	2.04 ± 0.15	2.12 ± 0.18	1.707	0.257
CRP (mg/L)	4.58 ± 0.85	6.84 ± 1.02	8.511	0.000
D-D (ng/mL)	235.68 ± 25.47	241.35 ± 26.77	0.767	0.485
FIB (g/L)	4.05 ± 0.56	5.02 ± 0.58	6.016	0.000
BNP (ng/L)	782.36 ± 50.19	2054.39 ± 103.42	55.327	0.000
UA (*μ*mol/L)	301.54 ± 23.28	336.75 ± 25.16	5.136	0.000
Scr (*μ*mol/L)	78.94 ± 6.84	92.33 ± 7.51	6.591	0.000
ALB (g/L)	37.05 ± 4.06	30.14 ± 3.51	6.438	0.000
TC (mmol/L)	3.85 ± 0.84	4.01 ± 0.89	0.654	0.517
TG (mmol/L)	1.72 ± 0.34	1.68 ± 0.31	0.435	0.559
LDL-C (mmol/L)	2.51 ± 0.76	2.65 ± 0.79	0.639	0.508
HDL-C (mmol/L)	1.20 ± 0.28	1.10 ± 0.25	1.332	0.236
Hb (g/L)	132.19 ± 15.42	130.18 ± 14.63	0.473	0.523
WBC (×109/L)	7.15 ± 0.63	8.45 ± 0.73	6.741	0.000
NC (×109/L)	4.51 ± 0.48	7.11 ± 0.61	16.748	0.000

The article "To Analyze the Influencing Factors of Senile Coronary Heart Disease Patients Complicated with Frailty Syndrome" was retracted in 2023. Reasons: signs of a paper mill; suspected computer-generated content; unreliable results or conclusions; concerns about the data.

**Table 3:** Multivariate logistic regression analysis.

Factors	Β value	SE value	Wx^2^	*P* value	OR value	95% CI
Age	−0.55	0.61	0.45	0.51	0.62	0.28–2.67
BMI	−0.71	0.78	0.59	0.63	0.74	0.31–2.89
Diabetes	−0.40	0.58	0.41	0.48	0.57	0.21–2.34
Congestive heart failure	−0.48	0.60	0.43	0.49	0.60	0.25–2.42
Chronic renal insufficiency	−0.65	0.71	0.54	0.60	0.71	0.28–2.75
COPD	2.15	0.96	0.43	0.02	1.23	1.05–5.63
Tumor	1.56	0.83	0.45	0.01	1.15	1.02–5.43
Hyperuricemia	−0.61	0.68	0.52	0.55	0.64	0.30–2.57
Arrhythmia	−0.53	0.60	0.42	0.48	0.59	0.24–2.51
IL-6	2.62	0.99	0.48	0.02	2.05	1.86–6.34
CRP	1.69	0.95	0.51	0.02	2.31	2.05–7.14
FIB	−1.05	0.86	0.63	0.69	0.71	0.35–2.64
BNP	2.05	0.87	0.63	0.01	2.45	2.16–7.33
UA	−0.92	0.75	0.69	0.77	0.68	0.41–2.93
Scr	2.16	0.88	0.71	0.01	3.52	2.57–7.84
ALB	2.28	0.95	0.76	0.01	3.61	2.67–7.95
WBC	−0.86	0.70	0.63	0.83	0.78	0.40–2.86
Number of neutral cells	1.84	0.91	0.82	0.02	2.89	1.76–6.48

## Data Availability

The simulation experiment data used to support the findings of this study are available from the corresponding author upon request.
